RETRACTED

# Effect of supplemental parenteral nutrition on all-cause mortality in critically Ill adults: A meta-analysis and subgroup analysis

**DOI:** 10.3389/fnut.2022.897846

**Published:** 2022-08-22

**Authors:** Peng Li, ChunYan Zhong, ShiBin Qiao, JunJun Liu

**Affiliations:** ^1^National Center of Gerontology of National Health Commission, The Key Laboratory of Geriatrics, Chinese Academy of Medical Sciences, Beijing Institute of Geriatrics, Institute of Geriatric Medicine, Beijing Hospital, Beijing, China; ^2^Department of Intensive Care Unit, Peking University ShouGang Hospital, Beijing, China; ^3^Department of Cardiology, People’s Hospital of Rizhao, Rizhao, China; ^4^Department of Oncology, National Center of Gerontology, Chinese Academy of Medical Sciences, Institute of Geriatric Medicine, Beijing Hospital, Beijing, China

**Keywords:** supplemental parenteral nutrition, enteral nutrition, critically ill, mortality, meta-analysis

## Abstract

**Objective:**

Several observational studies have demonstrated that increased nutritional delivery by supplemental parenteral nutrition (SPN) plus enteral nutrition (EN) reduces the rate of all-cause mortality in critically ill patients. Therefore, we aimed to compare and evaluate the effect of SPN plus EN on all-cause mortality in critically ill adults.

**Methods:**

Randomized controlled trials were retrieved from PubMed, Embase, Google Scholar, Cochrane Library, and Sinomed (up to May 2021). Adults with severe illness treated with SPN plus EN or with EN alone were enrolled. The risk of bias was evaluated using the Newcastle–Ottawa scale, and a meta-analysis was conducted using Stata software. The primary outcome was all-cause mortality and was evaluated by pooled odds ratio (OR) with the fixed-effects model. Required information size was also calculated using trial sequential analysis.

**Results:**

We identified 10 randomized controlled trials, with a total of 6,908 patients. No significant differences in rate of all-cause mortality (OR = 0.96, 95% CI: 0.84–1.09, *P* = 0.518), intensive care unit (ICU) mortality (OR = 0.90, 95% CI: 0.75–1.07, *P* = 0.229), and hospital mortality (OR = 0.95, 95% CI: 0.82–1.10, *P* = 0.482) were found between the SPN plus EN and EN alone groups. SPN plus EN support was associated with a significantly decreased risk of infection (OR = 0.83, 95% CI: 0.74–0.93, *P* = 0.001), although the duration of mechanical ventilation [standardized mean difference (SMD) = − 0.20], length of hospital stay (SMD = 0.12), and ICU stay (SMD = − 0.57) were similar between the two groups (all *P* > 0.05). Meta-regression analyses showed no significant correlations between all-cause mortality and baseline clinical factors, including patients’ age, the Acute Physiology and Chronic Health Evaluation II (APACHE II) score, time of SPN initiation, and follow-up duration (all *P* > 0.05). Subgroup analysis showed that SPN plus EN support was associated with a trend toward decreased rate of all-cause mortality in studies with follow-up < 30 days (OR = 0.61, 95% CI: 0.36–1.02, *P* = 0.058). Trial sequence analysis showed that the required information size for all-cause mortality was 16,972, and the cumulative Z-curve indicated no significant differences in the risk of all-cause mortality between the two groups (*P* > 0.05).

RETRACTED

**Conclusion:**

SPN plus EN support can significantly reduce the risk of infection, although it has no significant effect on all-cause mortality among critically ill patients. More studies are warranted to confirm these findings.

## Introduction

The incidence of malnutrition is high in critically ill patients. Critical illness is often associated with loss of appetite, inability to eat normally, proneness to severe nutritional deficiencies, muscle wasting, weakness, delayed recovery, increased risk of infection, prolonged hospital stay, and even high mortality (1–3). Artificial nutritional support can improve the nutritional status of critically ill patients, and enteral nutrition (EN) and parenteral nutrition (PN) are commonly used for clinical nutritional support. EN is the current nutritional support strategy. Early EN can protect intestinal function and maintain intestinal structure. At present, most people agree that EN can reduce infection and intensive care unit (ICU) stay and improve prognosis (4–6). However, patients with a severe illness often have gastrointestinal dysfunction or poor adaptation that results in inadequate feeding, which can affect nutritional status, increase the duration of infection and ICU stay, and risk of death (7).

Supplemental PN (SPN) refers to a mixed nutritional support method, in which part of the energy and protein is supplemented by PN when EN is insufficient (8, 9). Studies have found that reasonable SPN can meet the energy and protein needs of critically ill patients, promote protein synthesis, adjust nitrogen balance, improve nutritional status, and even reduce complications and improve prognosis (10). SPN also has a risk of causing overfeeding, hyperglycemia, liver dysfunction, prolonged mechanical ventilation, and infection (11). However, a recent retrospective cohort study with 182 patients with lung cancer showed that early SPN (within 72 h of development of granulocytopenia) significantly reduced the incidence of infection (*P* < 0.05) (12). In a meta-analysis, Alsharif et al. found that SPN plus EN significantly decreased the risk of nosocomial infection [relative risk (RR) = 0.733, *P* = 0.032] and ICU mortality (RR = 0.569, *P* = 0.030), although hospital mortality was comparable to that with EN alone (*P* > 0.05) (13). Therefore, there may be a survival benefit of early SPN among critically ill patients with malnutrition. However, several other studies have not shown a decreased risk of mortality with early SPN (*P* > 0.05) (14, 15). At present, the effect of early SPN on mortality has not been determined, and different countries or societies have different opinions on SPN recommendations (16–19). This study aimed to evaluate the impact of SPN plus EN support on the risk of all-cause mortality among critically ill adults.

RETRACTED

## Materials and methods

### Data sources and search strategies

We searched PubMed (January 2005 to May 2019), Embase (January 2005 to May 2021), Cochrane Library (up to May 2021), Google Scholar (up to May 2021)**, Sinomed** (up to May 2021), and ClinicalTrials.gov website (up to May 2021) using the terms supplemental parenteral nutrition (SPN), parenteral nutrition, EN, and critically ill. No language restrictions were applied. The review was registered at https://inplasy.com/inplasy-2022-7-0045/.

### Study selection

The inclusion criteria were as follows: (1) study type: published randomized controlled trials (RCTs); (2) study subjects: adult patients admitted for medical, surgical, or trauma diagnoses, and who stayed in the ICU for > 72 h; (3) intervention: the experimental group was given SPN plus EN support; (4) controls: control group was given EN support alone; and (5) outcome: the primary outcome was all-cause mortality. The exclusion criteria were as follows: (1) duplicate publications; (2) single-arm studies; (3) pediatric studies; and (4) case reports, animal studies, meeting reports, and reviews.

### Data collection

Two authors collected data using a standard data collection form about a year of publication, first author’s name, patient characteristics, treatment strategy, study quality, and primary and secondary outcomes. All the disagreements were resolved by discussion.

The literature was screened according to the Preferred Reporting Items for Systemic Reviews and Meta-Analyses (PRISMA) statement (20). The screening and data extraction of all the materials were independently completed by two reviewers and then cross-checked. When there were different opinions, they were discussed and resolved or other reviewers were consulted. The document selection process included: (1) Reading the title and abstract of the document; (2) screening all the possible relevant documents; and (3) extracting data, including study information, patient characteristics, study quality, intervention measures, and outcomes. The primary outcome was the risk of all-cause mortality. Secondary outcomes were rate of infection, mechanical ventilation duration, length of hospital stay, and ICU stay.

RETRACTED

### Quality evaluation

The PRISMA statement was followed for quality evaluation (20). Quality assessment was undertaken independently by two reviewers. We used the Newcastle–Ottawa Scale (NOS) to evaluate the methodological quality (21). The NOS varies from 0 to 9 and uses eight criteria that cover three components: patient selection, study group comparability, and outcomes assessment. Studies with the NOS score of ≥ 6 were considered high quality, and those studies with the NOS score of < 6 were considered low quality.

### Data synthesis and analysis

Data analysis was completed by three reviewers. Pooled odds ratio (OR) for dichotomous outcomes and standardized mean difference (SMD) for continuous outcomes were calculated with 95% CI. Heterogeneity was assessed by the *I*^2^ statistic and chi-squared test. *I*^2^ values of 25, 50, and 75% were considered as low, moderate, and high levels of heterogeneity, respectively (22). For outcomes with significant heterogeneity, the random-effects model was reported (22); for all the others, the fixed-effects model was reported (23).

Publication bias was tested using a funnel plot with Begg’s and Egger’s test (P for significant asymmetry < 0.1) (24, 25). The univariate meta-regression analysis was used to identify possible contributors to between-study variance. In particular, we investigated associations between the OR for mortality and clinically plausible factors, including patients’ age, the Acute Physiology and Chronic Health Evaluation II (APACHE II) score, time of SPN initiation, and follow-up duration. Sensitivity analysis was done by eliminating each study one at a time to evaluate the influence of each trial on the primary outcome and the robustness of the results (25).

All the analyses were performed according to the intention-to-treat principle. Statistical significance was set at 0.05 for the *Z*-test for OR. Results were analyzed quantitatively with STATA version 12.0 (StataCorp LP, College Station, Texas, United States).

### Subgroup analysis

On the basis of the mean level of baseline clinical data (patients’ age, the APACHE II score, time of SPN initiation, and follow-up duration), the studies were divided into those with age < 60.0 and ≥ 60.0 years, the APACHE II score < 20 and ≥ 20, early (≤ 72 h) and late (> 72 h) SPN initiation, and follow-up < 30 days and ≥ 30 days.

### Trial sequential analysis

In the meta-analyses, trial sequential analysis (TSA) was used to reduce the risk of reaching a false-negative conclusion (26). When the cumulative Z-curve crossed the trial sequential monitoring boundary or entered the futility area, a sufficient level of evidence for the anticipated intervention effect was reached, and no further trials were needed. If the Z-curve did not cross any of the boundaries and the required information size (RIS) had not been reached, evidence to reach a conclusion was insufficient, and more trials were needed to confirm the results. In this TSA for mortality, we estimated the RIS based on an OR reduction of 15%. The type I error (α) was 0.05 (two-sided) and the power (1–β) was 0.80. The control event proportion was 16.1% for all-cause mortality, which was calculated from the EN support group. The *I*^2^-value was 3.9%. The TSA was calculated using TSA version 0.9.5.10 beta.^1^

RETRACTED

## Results

### Search results

The process of study selection is shown in Figure 1. Initially, 1,305 potentially relevant articles were identified, and 41 articles were considered to be of interest after reviewing the titles and abstracts. After full-text review, 31 articles were excluded: 13 reviews, 11 incorrect comparisons, and seven with no clinical outcomes. Ultimately, 10 RCTs were included in the qualitative analysis and quantitative synthesis (Figure 1).

**FIGURE 1:** Sensitivity analysis of the impact of SPN and EN nutritional support treatment on all-cause mortality.

### Study characteristics and quality assessment

The 10 RCTs included (27–36) had a total of 6,908 patients. Most patients were critically ill and received mechanical ventilation. The mean age range was 40.1–77.5 years, and the mean follow-up ranged from 7 to 365 days. The time of SPN initiation was < 48 h in most studies. The average basic APACHE II score ranged from 17.0 to 25.0, and the average nutritional intake ranged from 14.2 to 28.0 kcal/kg/day. All the RCTs had the NOS score ≥ 8 and were, therefore, considered high quality. The results are shown in Table 1.

**TABLE 1:** Basic clinical characteristics of patients enrolled.

Trial	Year	Num.	Patients	Age (year)	SPN Treatment duration (day)	APACHE II score	SPN initiating time	Nutrition intake (kcal/kg/d)	Primary outcome	Follow (day)	NOS
Dunham et al. (27)	1994	10/12	Mechanically ventilated blunt trauma adult patients	NR	7	11.0/11.0*^a^*	24 h	2,153 KJ/2280 KJ	Mortality rate	28	8
Bauer et al. (28)	2000	60/60	Critically ill adult patients	53.0/55.0	4–7	43.0/41.0*^b^*	24 h	24.6/14.2	Levels of retinol-binding protein and prealbumin	90	9
Abrishami et al. (29)	2010	10/10	Critically ill adult patients	54.9/58.4	7	18.5/17.0	24 h	NR	Inflammatory indices	7	9
EPaNIC (30)	2011	2,312/2328	Critically ill adult patients had a score of 3 or more on NRS	64.3/63.8	16	23.0/23.0	3rd d	2,880 kcal	Number of ICU days and time to discharge from ICU	90	9
Heidegger et al. (31)	2013	153/152	Critically ill adult patients	61.0/60.0	5	22.0/23.0	4th d	28.0/20.0	Nosocomial infection rate	28	9
ANZICS (32)	2013	153/152	Critically ill adult patients	68.4/68.6	6	20.5/21.5	24 h	35 kcal/kg/d	All-cause mortality	60	9
Fan et al. (33)	2016	40/40	Severe traumatic brain injury	42.3/40.1	20	6–8*^a^*	48 h	105–126 KJ/kg/d	Immune function	28	9
Wischmeyer et al. (34)	2017	52/73	Adult patients with acute respiratory failure	55.8/55.1	7	20.5/20.8	24 h	1,641/1,272 kcal^§^	Rate of 30% improvement in nutrition delivery	60	9
Ridley et al. (35)	2018	51/49	Mechanically ventilated adults with at least one organ failure	59.0/60.0	7	18.0/19.0	24 h	1,892.0 kcal/1,298.0 kcal	Delivery of protein and energy	180	9
Bouleuc et al. (36)	2020	61/73	Advanced cancer à cachexia	66.6/66.2	NR	NR	< 48 h	30–35	Quality of life	NR	8

^§^Energy goals were reported as control 1,844 kcal, SPN 1,728 kcal) as were the amounts delivered for the first 7 days (control 69 ± 28, SPN 95 ± 13%), control 1,272 and SPN 1,641 kcal, respectively; *^a^*GCS score; *^b^*SAPS II score; num., number; SPN, supplemental parenteral nutrition; EN, enteral nutrition; NOS, Newcastle-Ottawa Scale; RCT, randomized controlled trial; NR, not reported.

RETRACTED

### Primary outcome

#### Risk of all-cause mortality

The 10 RCTs with a total of 6,908 patients reported all-cause mortality. Compared with the EN support group, SPN plus EN support was associated with a comparable risk of all-cause mortality (OR = 0.96, 95% CI: 0.84–1.09, *P* = 0.518). However, among studies with follow-up of 8–28 days, there was a trend toward decreased rate of all-cause mortality with SPN plus EN support (OR = 0.62, 95% CI: 0.36–1.04, *P* = 0.071) (Figure 2). Heterogeneity test showed no significant heterogeneity (*I*^2^ = 3.9%, *P* = 0.404). Neither the funnel plot nor Egger’s test (*P* = 0.86) suggested publication bias. Sensitivity analysis indicated that the removal of either study enrolled had no significant effect on the result. No significant differences in rate of ICU mortality (OR = 0.90, 95% CI: 0.75–1.07, *P* = 0.229) (Figure 3A) and hospital mortality (OR = 0.95, 95% CI: 0.82–1.10, *P* = 0.482) (Figure 3B) were found between the SPN plus EN and EN alone groups.

**FIGURE 2:** Effect of SPN and EN nutrition support treatment on all-cause mortality.

**FIGURE 3:** Effect of SPN and EN nutrition support treatment on ICU mortality **(A)** and hospital mortality **(B)**.

### Secondary outcomes

#### Rate of infection

Six studies reported infections in 6,633 critically ill patients. Overall, the rate of infection was significantly decreased in the SPN plus EN support group (OR = 0.83, 95% CI: 0.74–0.93, *P* = 0.001) (Figure 4). There was a low risk of heterogeneity (*I*^2^ = 26.4%, *P* = 0.236), and Egger’s test (*P* = 0.33) did not indicate publication bias. Sensitivity analysis indicated that the removal of either study enrolled had no significant effect on the result.

RETRACTED

**FIGURE 4:** Effect of SPN and EN nutrition support treatment on infection rate.

#### Mechanical ventilation duration

Seven RCTs reported the duration of mechanical ventilation. Compared with the EN alone group, SPN plus EN support was associated with a similar duration of mechanical ventilation (SMD = − 0.20, 95% CI: − 0.50 to 0.11, *P* = 0.215) (Supplementary Figure 1). There was significant heterogeneity (*I*^2^ = 93.9%, *P* = 0.000). Sensitivity analysis indicated that the removal of either study enrolled had no significant effect on the result.

#### Length of hospital stay

Eight studies reported the length of stay in ICU. Compared with the EN alone group, SPN plus EN support was associated with a similar length of ICU stay (SMD = − 0.57, 95% CI: − 1.63 to 0.50, *P* = 0.299), and there was significant heterogeneity (*I*^2^ = 99.5%, *P* = 0.000) (Supplementary Figure 2). Sensitivity analysis indicated that the removal of either study enrolled had no significant effect on the result.

Length of stay in hospital was also comparable between the two groups (SMD = 0.12, 95% CI: − 0.53 to 0.78, *P* = 0.708). There was a low risk of heterogeneity (*I*^2^ = 98.9%, *P* = 0.000) (Supplementary Figure 3). Sensitivity analysis indicated that the removal of either study enrolled had no significant effect on the result.

#### Meta-regression analyses

In meta-regression, no significant correlations were observed between the OR for mortality and mean age (*P* = 0.941), time of SPN initiation (*P* = 0.200), the APACHE II score (*P* = 0.924), and follow-up duration (*P* = 0.812) (Table 2).

**TABLE 2:** Meta-regression of baseline data and all-cause mortality.

Factors	β -coefficient	SE	95% CI	*P*
Mean age	0.002	0.021	–0.047 to 0.049	0.941
SPN initiating time	–0.288	0.324	–1.036 to 0.460	0.400
Follow-up	0.004	0.002	–0.003 to 0.004	0.812
APACHE II–	−0.002	0.023	–0.058 to 0.053	0.924

SPN, supplementary parenteral nutrition; APACHE, Acute Physiology and Chronic Health Evaluation; CI, confidence interval.

#### Subgroup analysis

In subgroup analysis, the pooled ORs for all-cause mortality in studies enrolling patients aged ≥ 60 years (OR = 0.96), with the lower APACHE II score (< 20) (OR = 0.592), or with early initiation of SPN (≤ 72 h) (OR = 0.98) were all similar to those in studies enrolling patients aged < 60 years (OR = 0.94), with the higher APACHE II score (≥ 20) (OR = 0.97), or with late initiation of SPN (> 72 h) (OR = 0.71). However, SPN plus EN support was associated with a trend toward decreased rate of all-cause mortality in studies with follow-up < 30 days (OR = 0.61, 95% CI: 0.36–1.02, *P* = 0.058) (Table 3).

RETRACTED

**TABLE 3:** Subgroup analysis of all-cause mortality.

Subgroup	Study num.	*I* ^2^	OR	95%CI	*P*
Mean age					
< 60 years	6	32.4%	0.94	0.62–1.42	0.756
≥ 60 years	4	0	0.96	0.83–1.11	0.564
APACHE II score					
< 20	5	45.3%	0.92	0.73–1.17	0.497
≥ 20	5	0	0.97	0.83–1.15	0.752
Early vs. late SPN					
Early SPN	8	9.5%	0.98	0.85–1.13	0.776
Late SPN	2	0	0.71	0.43–1.16	0.175
Follow-up duration					
< 30 Days	4	35.1%	0.61	0.36–1.02	0.058
≥ 30 Days	6	0	0.99	0.86–1.14	0.887

RCT, randomized controlled trial; SPN, supplementary parenteral nutrition; APACHE, Acute Physiology and Chronic Health Evaluation; OR, odds ratio; CI, confidence interval.

#### Trial sequential analysis

Trial sequential analysis showed that assuming a 15% difference in risk of all-cause mortality between the SPN plus EN and EN alone groups, the RIS required 16,972 participants. The cumulative Z-curve did not cross-trial sequential boundaries, indicating non-significant differences in the risk of all-cause mortality between the groups. Therefore, SPN plus EN support had no significant effect on all-cause mortality among critically ill patients (*P* > 0.05) (Supplementary Figure 4).

## Discussion

This meta-analysis, including all the available evidence, showed that the application of SPN plus EN did not significantly decrease the risk of all-cause mortality among critically ill patients (OR = 0.96), although there was a trend toward decreased rate of all-cause mortality in studies with follow-up < 30 days (OR = 0.61).

The guidelines of the American Association for Parenteral and EN, the European Association for Parenteral and EN, and the SPN Chinese Expert Consensus all indicate that when EN alone cannot meet the energy and protein needs of patients, SPN provides the extra energy and protein to meet the body’s target needs and avoid the risk of malnutrition (16–19). Meanwhile, proper SPN can reduce the initial amount of EN and reduce the related risk of diarrhea and vomiting (16–19).

SPN may improve the prognosis and reduce the risk of infection in critically ill patients. The ANZICS study involving 1,372 critically ill adults with contraindications to early EN found that early PN within 24 h of ICU admission significantly reduced invasive mechanical ventilation time from 7.73 to 7.26 days (*P* = 0.01) (32). Another study of 305 critically ill subjects found that the incidence of nosocomial infections in patients with SPN was significantly lower than in patients with EN nutritional support alone, and the duration of antibiotic use was reduced (31). Combining five randomized clinical studies, Alsharif et al. indicated that compared with EN alone, SPN + EN decreased the risk of nosocomial infections (RR = 0.733, *P* = 0.032) and ICU mortality (RR = 0.569, *P* = 0.030). No significant differences were observed between the two groups in the length of hospital and ICU stay, hospital mortality, and duration of mechanical ventilation (all *P* > 0.05) (13). However, several studies showed that, for critically ill patients with high malnutrition risk, inadequate calorie supplementation after gastrointestinal surgery was associated with increased 30-day mortality in patients with high malnutrition, and adequate caloric or protein supply with SPN had a better survival benefit (37). Similarly, Sim et al. found that baseline malnutrition status was associated with the survival benefit of SPN, which was significant in patients with high malnutrition risk and non-significant among those with low malnutrition (38). Similar to previous studies (39, 40), our meta-analysis of 6,908 critically ill patients from 10 RCTs demonstrated that SPN plus EN significantly reduced the risk of infection, but had no significant effect on all-cause mortality and duration of mechanical ventilation and hospital stay.

RETRACTED

The timing of SPN initiation is still controversial. The results of a multimedium RCT clinical study showed that early PN (day 4) significantly reduced the infection rate and use of antibiotics in severely ill patients (31). However, the Early Parenteral Nutrition Completing EN in Adult Critically Ill Patients (EPaNIC) study (30) showed that late PN (day 8) reduced the risk of complications, shortened mechanical ventilation time, and decreased hospitalization costs compared with early SPN (within 48 h). The rate of being discharged alive from the ICU [hazards ratio (HR) = 1.06, *P* = 0.04] and from the hospital (HR = 1.06, *P* = 0.04) was higher in the late SPN group (40). Heyland et al. found that early SPN increased the risk of nosocomial infections and significantly lengthened ICU stay (*P* < 0.05) (41). For critically ill children, the Pediatric Early vs. Late Parenteral Nutrition in ICU (PEPaNIC) study showed that early initiation of PN significantly increased nosocomial infection rate, mechanical ventilation time, and ICU stay (*P* < 0.05) (42). In a recent cohort study, 317 patients undergoing emergency abdominal surgery for severe infection were divided into low (*n* = 206) and high (*n* = 111) malnutrition risk according to the modified Nutrition Risk in Critically ill (mNUTRIC) score and body mass index (BMI) (37). Furthermore, all were subdivided into the early SPN group (within 48 h) and the control group (who did not receive PN). The authors found no significant difference in mortality among the low malnutrition risk patients (*P* > 0.05). However, among those with high malnutrition risk, the early SPN group had significantly increased caloric adequacy (0.88 vs. 0.60) and protein amounts (0.94 vs. 0.47 g/kg) (37). The risk of 30-day mortality (7.6 vs. 26.7%, *P* = 0.006) and in-hospital mortality (13.6 vs. 28.9%, *P* = 0.048) was also significantly lower in the early SPN group than in the control group (37). Similar to previous studies, we found that early SPN lowered the risk of mortality among critically ill patients (OR, 0.62; 95% CI: 0.43–0.90), especially among aged subjects with high malnutrition risk. However, more RCTs are needed to confirm these findings. We suggest that for adults with high nutritional risk (NRS-2002 ≥ 5 or the NUTRIC score ≥ 6), if EN does not reach 60% of target energy and protein requirements within 2–3 days, early SPN is recommended. Therefore, although the timing of SPN is still controversial in the clinic, according to the patient’s condition, an individualized nutritional support regimen should be administered to balance the risks and benefits.

RETRACTED

The ratio of PN solutions may affect prognosis. The PEPaNIC study indicated that increasing the dose of amino acids added early increased infection rate and decreased survival rate. Increased doses of glucose and fat were independent factors for early pediatric ICU (PICU) survival (43). Previous studies have confirmed that the amount of calories can also affect prognosis (44, 45). However, without individual patient data, we could not evaluate these findings. Therefore, more research is needed to evaluate the effect of PN formulation ratio, and calorie and protein intake pathways on prognosis.

Four updated meta-analyses and systematic reviews of EN plus SPN in critically ill patients were recently published (13, 39, 40, 46). Lewis et al. performed a meta-analysis of 8,816 critically ill subjects (trauma, emergency, and postsurgical patients) from 23 RCTs and two quasi-RCTs. They found insufficient evidence to determine whether EN is better or worse than PN or combined EN and PN for in-hospital mortality at 90 and 180 days, and the number of ventilator-free days and adverse events (46). Another meta-analysis conducted by Fuentes et al. had a similar conclusion (40). In our previous study, we confirmed that SPN plus EN support decreased the infection rate of critically ill patients in ICU, but it had no obvious influence on overall all-cause mortality (39). However, in a recently published meta-analysis (13), Alsharif et al. indicated that compared with EN alone, SPN + EN decreased the risk of ICU mortality (RR = 0.569, *P* = 0.030). They searched RCTs published in the English language from January 1990 to January 2019 and five RCTs were included. Several important and well-known clinical trials were not included in their study, such as the EPaNIC (30) and ANZICS (32). They only included studies published in English, which could also have increased the risk of heterogeneity. The included RCTs had different categories of ICU patients (burn, trauma, and others), and the responses to nutritional support were different in each category. Moreover, several confounding factors, including the type of enteral formula used, the form of lipids used in the PN solution, and equations used to estimate the energy requirement, could have interfered with the effects of SPN plus EN support. Additionally, there was a risk of overfeeding. Although the target energy intake seemed similar between the studies, it was not individualized based on each patient’s needs. In our updated meta-analysis and systematic review, rates of all-cause mortality, ICU mortality, and hospital mortality were comparable between the SPN plus EN and EN alone groups (*P* < 0.05). This was in line with previous studies (39, 40, 46). Furthermore, although SPN plus EN support was associated with a significantly decreased risk of infection, more large, multicenter randomized clinical studies with rigorous methodology are warranted to confirm these findings (47).

RETRACTED

### Limitations

Our study had several limitations: (1) our meta-analysis was based on study-level data with the flaws of the original studies; (2) two studies were cohort studies, with an increased risk of heterogeneity. Therefore, the overall outcome may have been affected; (3) There was a risk of geographical variations. All the 10 studies had small differences in the patients’ characteristics, conditions, SPN treatment strategies, and follow-up periods; and (4) the sample size was small. TSA showed that, assuming a 15% difference in the risk of all-cause mortality between the SPN plus EN and EN alone groups, the RIS required 16,972 participants, and the accrued information size was only 6,908. Therefore, larger clinical studies are needed to evaluate the benefits of SPN plus EN support for critically ill patients.

## Conclusion

The results show that SPN plus EN can lower the rate of infection among critically ill patients. However, it has no significant effect on all-cause mortality and length of hospital stay. As a result of the small sample size of the RCTs included in this study, more studies are needed to confirm these findings.

RETRACTED

## Data availability statement

The raw data supporting the conclusions of this article will be made available from the corresponding author by request.

## Ethics statement

Ethical review and approval were not required for the study on human participants in accordance with the local legislation and institutional requirements. Written informed consent for participation was not required for this study in accordance with the national legislation and the institutional requirements.

## Author contributions

PL wrote the main manuscript text. CZ and SQ analyzed the data. JL designed the work. All authors contributed to the article and approved the submitted version.

## Footnotes

1
www.ctu.dk/tsa

## Supplementary material

Supplementary Figure 1 Flow diagram.

Supplementary Figure 2 Effect of SPN and EN nutritional support treatment on mortality.

Supplementary Figure 3 Subgroup analysis of mortality in different subsets.

Supplementary Figure 4 Trial sequential analysis.
